The article "Visual Mechanism Characteristics of Static Painting Based on PSO-BP Neural Network" was retracted in 2023. Reasons: unreliable results or conclusions; concerns about the data; concerns about the peer review; concerns about the citations.

# Visual Mechanism Characteristics of Static Painting Based on PSO-BP Neural Network

**DOI:** 10.1155/2021/3835083

**Published:** 2021-08-09

**Authors:** Hai Wang, Hongtao Zhang

**Affiliations:** ^1^School of Architectrual and Artistic Design, Henan Polytechnic University, Jiaozuo, Henan 454003, China; ^2^Shool of Foreign Studies, Henan Polytechnic University, Jiaozuo, Henan 454003, China

## Abstract

Static painting works have independent theme significance in the framework of Chinese painting history, and their overall structure, lightness structure, and color structure all show different characteristics of visual mechanism. In order to extract the visual mechanism features effectively, this experiment uses the PSO algorithm to optimize the BP neural network, constructs the PSO-BP neural network for feature recognition and extraction, and compares it with the training results of other algorithms. The results show that the prediction accuracy, recognition accuracy, and ROC curve of PSO-BP neural network are high, which shows that the convergence of PSO-BP neural network is good, and it can effectively complete the recognition and analysis of people and effectively extract the visual mechanism features of static writing paintings.

## 1. Introduction

In the process of appreciation and analysis of static painting works, perception has certain limitations only through the human eye, so it is very important to extract the visual mechanism features with the help of relevant algorithms. Gu et al. [1] believed that the grinding process of SiCp/AI composite can provide certain guidance for energy saving and consumption reduction. By applying the PSO-BP neural network prediction model to the prediction of grinding energy consumption of the material, it is successfully found that the model constructed by PSO-BP neural network has high prediction accuracy. Ma et al. [2] applied BP neural network prediction model to the analysis of heat transfer coefficient in view of the determination of heat transfer coefficient in the range of supercritical water pressure. The experimental results show that there are small errors in specific heat, mass flow, heat flow, pressure, and diameter, and the prediction effect of BP neural network prediction model is better. Wang et al. [3] constructed the prediction model of wind farm range based on BP neural network, optimized it with PSO algorithm, and successfully realized the prediction of output power interval.

Jian et al. [4] believed that fractional ladder calculus can be used for information processing and modeling. In order to improve its performance, BP neural network is used for optimization and simulation analysis, which has successfully improved its learning efficiency. In the work of Lü et al. [5], using LM-BP neural network to simulate the experimental results of shear wave in hinge strata under different axial pressure and other states, it is found that LM-BP neural network can be widely used in S-wave velocity fitting under multiple working conditions. He and Zhang [6] put forward a two-stage mixed method to predict the phosphorus content of molten steel at the end point of converter steelmaking. The weighted K-means is used to generate clusters with homogeneous data, and the fuzzy neural network is used to obtain accurate prediction results. Li et al. [7] combined chaos algorithm with CGA to improve the real-time performance and accuracy of gesture recognition, aiming at the shortcomings of easily falling into local minima and slow convergence speed of BP neural network in gesture recognition. Aiming at the problem that the traditional copula model cannot deal with the real-time data required for fault prediction, Luo et al. [8] combined BP neural network and copula and verified the effectiveness of the combined model. Wang et al. [9] used normalized data and BP neural network to study the classification of pulse signal and the selection of characteristic factors based on BP neural network classification method and found that the less influence factors, the worse the effect.

Wu et al. [10] used GA to improve BP neural network, which solved the problems of slow convergence speed and easiness to fall into local minimum when BP neural network was applied to land ecological security evaluation alone. Geng et al. [11] added *k*-fold cross validation method to BP artificial neural network model, which successfully verified the effectiveness of the model in SOC estimation of lithium battery. Liu and Yin [12] believed that the traditional BP neural network has the disadvantages of slow convergence speed and low accuracy, which is easy to fall into local minimum. Therefore, this paper proposes an improved PSO algorithm to improve its application effect. Aiming at the problem of wave height prediction, Wang et al. [13] combined the hybrid thinking evolutionary algorithm with BP neural network and verified that MEA-BP algorithm has high operation efficiency and prediction accuracy [13].

To sum up, BP neural network and PSO neural network have their own advantages, which can carry out high-precision model prediction in different fields. The organic combination of the two can significantly improve the quality of the prediction effect. In view of this, this experiment uses PSO-BP neural network to explore the extraction of visual mechanism features of static writing paintings in order to achieve comprehensive and efficient feature recognition and extraction.

## 2. Image Preprocessing of Visual Mechanism Characteristics of Static Writing Paintings

### 2.1. Image Gray Processing of Static Writing Paintings

The main reason why the visual mechanism features of static writing paintings are different from the extraction process of other image visual features is that the static writing paintings are in the two-dimensional state, which are different from the three-dimensional images directly recognized by human eyes. However, when extracting the visual mechanism features of static painting works, the main principles and processes are still similar, as shown in Figure 1.

It can be seen from Figure 1 that the feature extraction of visual mechanism of static writing painting image is mainly divided into two stages, namely, the training attribute model stage and the attribute feature extraction stage, which are realized by means of feature extraction, attribute modeling, model prediction, and so forth. Then, the work image is grayed, and the color image is quickly converted into gray image to ensure the timeliness and effectiveness of image processing [14–17]. Image graying based on weighted average is an effective image processing method, and the calculation formula is shown as follows:

(1) $$\begin{array}{c} F\left(i,j\right)=aR\left(i,j\right)+bG\left(i,j\right)+cB\left(i,j\right), \end{array}$$

where (*i*, *j*) represents the image pixel coordinate position; *a*, *b*, and *c* all represent the weighting coefficients of gray-scale processing, and their values are usually 0.3, 0.59, and 0.11, respectively. The gray values of all pixels in the image to be processed are defined as (2) and (3) for details.

(2) $$\begin{array}{c} Gray=0.3R\left(i,j\right)+0.59G\left(i,j\right)+0.11B\left(i,j\right), \end{array}$$

(3) $$\begin{array}{c} R=G=B=\text{Gray}. \end{array}$$

In the above formula, *R* represents the red component in the pixel of the image to be processed; *G* stands for green, that is, the green component in the image pixel; similarly, *B* represents the blue component in the target image pixels [18]. The threshold value of foreground and background of the image to be detected is set to *T*, so that the average value of gray level is *u*; the proportion of foreground points in the whole image is *w*_0_, and the average gray value is *u*_0_; the proportion of background points is *w*_1_, and the corresponding average gray value is *u*_1_; if the variance between classes is expressed as *g*, we can get the two following formulas:

(4) $$\begin{array}{c} u=w_{0}\times u_{0}+w_{1}\times u_{1}, \end{array}$$

(5) $$\begin{array}{c} g=w_{0}\times {\left(u_{0}-u\right)}^{2}+w_{1}\times {\left(u_{1}-u\right)}^{2}. \end{array}$$

The simultaneous formula (4) and formula (5) have the following formula:

(6) $$\begin{array}{c} g=w_{0}\times w_{1}\times {\left(u_{0}-u_{1}\right)}^{2}. \end{array}$$

According to equation (6), when the difference between the foreground and background of the image to be detected is maximized, *g* can reach the maximum value, and *T* can reach the optimal threshold at this time.

### 2.2. Image Feature Extraction of Static Painting Works

In the static painting works, the objects in the painting works are usually composed of the same gray area and texture. When the vision perceives the image, it usually extracts the image region by segmenting the image edge; then the image is segmented and understood semantically, and the information is refined and analyzed [19]. The image is mainly divided according to the information level. The low-frequency signal can reflect the scale strength of the image and can describe its shape and position by showing the flatness of the image. This part is the intensity synthesis layer. High-frequency signal reflects the details and edge information in the image, highlighting the information that has changed dramatically. This part is called contour detail layer [20]. The dense information in the image feature space of static painting works needs to be obtained under the action of algorithms, especially kernel function, which can effectively estimate the kernel density of the image. In this experiment, Gaussian kernel function with symmetry is used to smooth the image. See the following equation for details:

(7) $$\begin{array}{c} K\left(x\right)=\frac{1}{\sqrt{2\pi \sigma^{2}}}\exp\left(-\frac{x^{2}}{2\sigma^{2}}\right). \end{array}$$

According to the kernel function *K* in equation (7) and the bandwidth parameter *h*, the probability density of the target image can be estimated, as shown in the following equation:

(8) $$\begin{array}{c} f\left(x\right)=\frac{1}{nh^{d}}\sum_{i=1}^{n}K\left(\frac{x-x_{i}}{h}\right). \end{array}$$

In the above equation, *n* represents the number of pieces of data in the image. Set *a*_*i*_ as the existing pixel, and *i* satisfies *i*=1,2,…, *n*. When *a*_*i*_ is taken as the center of the circle with radius *h*, all the points in this range are represented as *x*_*i*_. If *a*_*i*_ and *x*_*i*_ have high similarity color values, it can be judged that they have high probability density, and the probability density is positively correlated with the adjacent degree of their positions. Therefore, Gaussian kernel function can provide strong support for image information extraction and scale transformation. By subtracting the original image from the high-frequency edge image, the texture contour information of the image can be obtained. The flowchart is shown in Figure 2.

After the static painting image is input, the Gaussian kernel function is used to smooth the image. Then, the high-frequency feature texture information in the target image can be effectively extracted under the effect of Gaussian pyramid scale transformation, and the complete image texture image can be finally output.

## 3. Construction of Image Classification Model Based on PSO-BP Neural Network

### 3.1. Structure and Composition of BP Neural Network

The extraction of visual mechanism features of static writing paintings depends on the image processing and image analysis advantages of artificial neural network. Backpropagation (BP) neural network, as one of the classic feedforward neural networks, has stronger adaptive ability and learning ability [21–23]. Under the effect of error backpropagation, BP neural network can continuously adjust the training network until the best network model is retained, and its basic component is neuron [24, 25]. Multiple neurons can form a complete basic network layer under the effect of full connection; multiple basic network layers interact to form a network structure layer.

The most common three-layer structure of BP neural network is that including input layer, hidden layer, and output layer. There is nonlinear mapping relationship between each network layer. The input layer contains multiple vectors, expressed as *x*=(*x*_1_, *x*_2_,…, *x*_*n*_), while the output layer contains *y*=(*y*_1_, *y*_2_,…, *y*_*n*_) vectors. Between the input layer and the hidden layer and between the hidden layer and the output layer, there are connection weights, which are expressed as *w*_*ij*_ and *t*_*jk*_, respectively. The network layer is also covered with four modules, which are used to complete the input and output of nodes, function activation, error calculation, and self-learning [26, 27]. The node input and output module means that, in the process of network training, the image data is transferred layer by layer under the function operation. The activation of the function means that the data of the upper network node is transferred to the lower network under the action of nonlinear transformation. In the error calculation module, there is a certain difference between the actual output and the expected output of the network node. The square statistical result of the difference is recorded as the error value. The error value is the difference between the actual output and the expected output, which can directly reflect the advantages and disadvantages of the network performance. The calculation formula is shown in the following equation:

(9) $$\begin{array}{c} e_{p}=\frac{1}{2}\sum_{k=1}^{m}{\left(y_{k}-{\hat{y}}_{k}\right)}^{2}. \end{array}$$

In the above equation, the values of actual output and expected output are represented, respectively.

The self-learning module undertakes the self-learning task of BP neural network. By continuously updating and connecting the weights of each network layer in the process of network training, it can effectively match the input and output data features and finally achieve accurate classification. The weight correction formula of network training is expressed as follows:

(10) $$\begin{array}{c} \Delta w_{ij}\left(i+1\right)=\eta \Phi_{i}{Ο}_{j}+\partial \Delta \;w_{ij}\left(n\right). \end{array}$$

In the above equation, *η* and ∂ represent the learning factor and momentum factor in the module, respectively; Φ_*i*_ represents the calculation error at the output node *i*; and Ο_*j*_ represents the output value at the output node *j*.

### 3.2. PSO Algorithm Optimization and Its Implementation Process

Because of the randomness of BP neural network in initializing the weights, it often shows instability when it is applied to image classification and recognition. Therefore, optimizing the initial value can help to ensure the reliability of the network. As an intelligent stochastic optimization algorithm, particle swarm optimization (PSO) can play a more significant optimization utility [28–30]. PSO algorithm originated from the process of birds' predation, which has strong global optimization ability. The algorithm uses the cooperation and competition between particles to complete the search. By constantly adjusting the speed, position, and fitness of particles, it can effectively achieve global optimization. According to the constant change of particle velocity and position, PSO algorithm can get the optimal position of particle extremum, which includes the extremum of individual and group [23, 24]. If there is a *d*-dimensional particle swarm space in the network training, the change of velocity in the updating process can be expressed as follows:

(11) $$\begin{array}{c} V_{i\;d}^{k+1}=\omega V_{i\;d}^{k}+c_{1}r_{1}\left(P_{i\;d}^{k}-X_{i\;d}^{k}\right)+c_{2}r_{2}\left(P_{g\;d}^{k}-X_{g\;d}^{k}\right). \end{array}$$

In the above equation, *k*is the number of iterations in network training, *ω* is the inertia weight, *V* is the speed of particle update, *X* is the location of particle update, *X*_*i*_=(*x*_*i*1_, *x*_*i*2_,…, *x*_*i*  *D*_) is the potential solution, and *V*_*i*_=(*V*_*i*1_, *V*_*i*2_,…,*V*_*i*  *D*_)^*T*^ is the corresponding speed, while *P*_*i*_=(*P*_*i*1_, *P*_*i*2_,…,*P*_*i*  *D*_)^*T*^ and *P*_*g*_=(*P*_*g*1_, *P*_*g*2_,…,*P*_*g*  *D*_)^*T*^ scale represent the individual extreme value and group extreme value, respectively, *c*_1_ and *c*_2_ are nonnegative acceleration constants, and *r*_1_ and *r*_2_ are values obtained in the interval. The position change of particle update is shown in the following equation:

(12) $$\begin{array}{c} X_{i\;d}^{k+1}=X_{i\;d}^{k}+V_{i\;d}^{k+1}. \end{array}$$

According to equation (11) and equation (12), the implementation process of PSO algorithm can be summarized, as shown in Figure 3.

In the process of PSO algorithm implementation, we need to initialize the velocity and position of all the particles in PSO firstly. Then the fitness value of each particle is calculated. The individual extremum was obtained and compared with fitness value to complete the optimization of individual extremum. Then, the population extremum is optimized, and the fitness value is compared with the current population extremum. The velocity and position of particles are updated continuously. Finally, it is judged whether the fitness value meets the expected requirements. If not, it is circularly processed to find the optimal fitness value until the optimal value is obtained. In this process, there are four types of fitness functions which need to be applied, as shown in Figure 4.

Figure 4(a) shows the three-dimensional realization of Ackley function, which includes a large number of local minimum points. It can be seen that there is a minimum value of the function, and its abscissa and ordinate are all 0. Therefore, the function is usually used in the optimization of extreme points. The Ackley function can be expressed as follows:

(13) $$\begin{array}{c} f_{1}\left(x\right)=-c_{1}\exp\left[-0.2\sqrt{\frac{1}{n}\sum_{j=1}^{n}x_{j}^{2}}\right]-\exp\left(\frac{1}{n}\sum_{j=1}^{n}\cos\left(2\pi x_{j}\right)\right)+c_{1}+e. \end{array}$$

Figure 4(b) shows the Schaffer function, in which there are uncountable maximum and minimum points, the maximum value is 1, and the abscissa and ordinate values of the maximum point are 0. This function is only a fitness function, which is usually not applied to the test of global optimization ability. The function expression is shown in the following equation:

(14) $$\begin{array}{c} f_{2}\left(x\right)=0.5-\frac{\sin\left(\sqrt{x^{2}+y^{2}}\right)-0.5}{{\left[1+10^{-2}\left(x^{2}+y^{2}\right)\right]}^{2}}. \end{array}$$

Figure 4(c) shows the three-dimensional implementation of the Rastrigin function, which contains many local extremums and can be used as one of the test functions for global optimization ability. See the following equation for details of the function:

(15) $$\begin{array}{c} f_{3}\left(x\right)=\sum_{i=1}^{n}\left(x_{1}^{2}-10\;\cos\left(2\pi x_{1}\right)+10\right). \end{array}$$

Figure 4(d) shows Rosenbrock function, which is a nonconvex function. It is difficult to get the minimum value. It can be applied to the evaluation of the algorithm to judge whether it has the ability to avoid premature phenomenon. The following equation shows the expression of Rosenbrock function:

(16) $$\begin{array}{c} f_{4}\left(x\right)=\sum_{i=1}^{n}\left[{\left(100\left(x_{i+1}-x_{i}^{2}\right)\right)}^{2}+{\left(x_{i}-1\right)}^{2}\right]. \end{array}$$

### 3.3. PSO-BP Algorithm Process and Model Construction

According to the above content, BP neural network has great randomness in determining the initial weights of the network, and PSO algorithm has a significant advantage in network weight optimization. Therefore, this experiment organically combines the two algorithms to construct the PSO-BP neural network model. PSO-BP neural network can effectively use the PSO algorithm to update the particle extreme value so as to avoid the risk of BP neural network due to the randomization of initial value. The algorithm implementation process is shown in Figure 5.

Observing Figure 5, it can be found that the PSO-BP neural network algorithm is mainly divided into two parts: BP neural network and PSO algorithm, which are independent of each other and work together. Firstly, the structure and related parameters of BP neural network need to be initialized, and then the weight vector *W* is constructed by combining with its connection weights, and *W* is used as the space particle in PSO algorithm. The parameters of PSO, including inertia weight, acceleration constant, particle velocity, and particle position, are set, and the velocity and position are updated continuously. By calculating and iterating the fitness values of all particles in the space, the new fitness function values of particles can be obtained, and then the optimal extremum, including individual extremum and group extremum, can be selected by comparing before and after. The fitness function is usually represented by the mean square error of BP neural network in the process of network training. The following formula is the calculation formula of fitness function:

(17) $$\begin{array}{c} E\left(x_{p}\right)=\frac{1}{N}\sum_{p=1}^{n}\sum_{k=0}^{m}{\left(y_{pk}\left(x_{p}\right)-t_{pk}\right)}^{2}. \end{array}$$

In the above equation, *x*_*p*_ represents the *p*-th group of input samples, and *p* meets the requirements of *p*=1,2,…, *n*; *y*_*pk*_ is the *k*th output result of *x*_*p*_, *t*_*pk*_ is the *k*th output expected value of *x*_*p*_, and *k* satisfies *k*=1,2,…, *m*. After that, the weight can be optimized. If the optimal value of fitness function obtained is better than the preset value or the number of iterations reaches the maximum, the global optimal weight *w*_*sq*_ has been obtained. Then the error is calculated and adjusted, and the new weights are used for comparison and calculation. When the error meets the requirements, the network training can be terminated.

## 4. Experimental Results and Analysis

### 4.1. Subjective Evaluation Results of PSO-BP Algorithm

In this experiment, PSO-BP algorithm is applied to the analysis of static painting works. Firstly, the target image is grayed to provide support for the later extraction of visual mechanism features. The results are shown in Figure 6.

Figure 6(a) shows the original picture of the static object painting works selected in this experiment. This picture presents a relatively rich color. Each single element in the picture is on the paper. Dragonfly, loquat, bamboo basket, signature, and seal have different color performance. In view of this, it is difficult to extract and analyze the features of its visual mechanism, so the corresponding image preprocessing operation is needed.  Figure 6(b) shows the image presented after gray-scale processing of the static writing painting by applying PSO-BP algorithm. Compared with Figure 6(a), the gray-scale image is helpful for the extraction of image features or object detection in the later stage and can improve the recognition accuracy and processing efficiency of image visual mechanism features to a certain extent.  Figure 6(b) shows that the PSO-BP algorithm can comprehensively extract the shape feature, texture feature, and color feature components of the target image when extracting the visual mechanism features of the target image, which provides an accurate basis for the prediction and classification of the target image.

### 4.2. Comparison of Objective Evaluation Results between PSO-BP and Other Algorithms

In order to explore the effectiveness and accuracy of PSO-BP neural network in extracting the visual mechanism features of static writing paintings from the objective level, this experiment selected 100 static writing paintings as a complete training sample and conducted 3000 iterations in batches. In the iterative training process of each batch of training samples, the average accuracy of training samples and other data are calculated and recorded, and the results are plotted as shown in Figure 7.

According to Figure 7, at the beginning of network training model, the initial value of loss function is larger, about 1.77, but it shows a downward trend of cliff type. The recognition accuracy increased sharply from 0 to 0.75. When the training times reach 100, the decreasing trend of loss function value gradually slows down. The increase of recognition accuracy of the sample image is also reduced, and the accuracy reaches about 80%, which indicates that the model proposed by PSO-BP neural network can achieve better training effect. In the continuous process of network training, the change range of loss function value and recognition accuracy is small. When the number of training times reaches 500, the former value is still high, but it keeps a small decline trend, and the latter is close to 90%. When the network training is carried out 2000 times, the value of loss function almost does not decline and only has a small fluctuation. The recognition accuracy tends to be flat. In order to get the optimal training results and avoid the network training model falling into the local optimal state, the network model continues to train. When the number of training times reaches 3000, the loss function value and recognition accuracy do not show significant changes, and the difference range is within the normal error range. This shows that the model constructed by PSO-BP neural network algorithm has reached the ideal state, and the network training has ended smoothly. In addition, the PSO-BP algorithm proposed in this paper is compared with the general neural network algorithm in recognition accuracy. The results are shown in Figure 8.

As can be seen from Figure 8, the recognition accuracy of PSO-BP algorithm is higher for static painting samples. When the training times are less than 100, the recognition accuracy of PSO-BP algorithm is significantly higher than that of ordinary neural network algorithm. When the training times is more than 100, the growth rate of recognition accuracy of the two algorithms decreases significantly, and the accuracy tends to be stable. In the whole process of network training, the recognition accuracy of PSO-BP algorithm is significantly higher than that of ordinary neural network algorithm, which means that the network training model constructed by the former has faster convergence speed, smaller oscillation level of recognition accuracy, and stronger stability of the model. In this experiment, a variety of neural network algorithms are selected for comparative analysis with PSO-BP neural network algorithm, and receiver operating characteristic (ROC) curves are compared. The results are shown in Figure 9.

In the ROC curve, TP is defined as the correct recognition part of the visual mechanism feature of the static writing painting, and FP is defined as the wrong recognition part. The ordinate axis and abscissa axis in Figure 9 represent true positive rate (TPR) and false positive rate (FPR), respectively, and Figure 9 clearly shows that the ROC curve of PSO-BP algorithm is always higher than those of the other eight algorithms. The comparison results of area under curve (AUC) value show that the AUC value of PSO-BP algorithm is higher than those of the other eight algorithms, which shows that PSO-BP can show superior detection and analysis effect in the recognition and detection of visual mechanism features of static writing paintings.

## 5. Conclusion

Static writing paintings are rich in unique artistic charm, and the extraction of their visual mechanism features has certain artistic value and practical significance. In order to accurately grasp the characteristics of their visual mechanism, this project uses PSO algorithm to optimize BP neural network, constructs the network prediction model of PSO-BP neural network, and applies it to the network training of work sample set. This is a new and complex improved neural network, which can significantly improve the prediction efficiency of the original BP neural network. The experimental results show that when the number of iterations reaches 3000, the recognition accuracy of the model is close to 100%, and the difference between the loss function value and the recognition accuracy is within the normal error range. The model constructed by PSO-BP neural network algorithm can quickly reach the ideal state, the convergence speed is extremely fast, the oscillation level of recognition accuracy is smaller, and the stability of the model is stronger. PSO-BP neural network can extract the visual mechanism features of static painting works comprehensively and effectively, which has high application value. Compared with other neural networks such as CNN, ANN, and FFNN, the PSO-BP neural network proposed in this paper has higher recognition rate and can provide strong support for effective feature extraction. Although PSO-BP neural network is successfully used to extract and analyze the visual mechanism features of static painting works, due to the space limitation, the subjective results of the work analyzed by PSO-BP neural network are not elaborated in detail, which is expected to be improved and expanded in the future research.

## Figures and Tables

**Figure 1:** Schematic diagram of image visual mechanism feature extraction process.

**Figure 2:** Extraction of texture information of static painting works.

**Figure 3:** Flowchart of PSO algorithm.

**Figure 4:** Three-dimensional diagram of four fitness functions. (a) Three-dimensional graph of Ackley function. (b) Three-dimensional graph of Schaffer function. (c) Three-dimensional graph of Rastrigin function. (d) Three-dimensional graph of Rosenbrock function.

**Figure 5:** Implementation process of PSO-BP neural network algorithm.

**Figure 6:** Static painting image before and after graying by PSO-BP algorithm. (a) The original picture of static painting. (b) Gray-scale image static painting.

**Figure 7:** Relationship between sample image recognition accuracy and training batch.

**Figure 8:** Comparison results of recognition accuracy between PSO-BP algorithm and common neural network algorithm.

**Figure 9:** Comparison of ROC curve between PSO-BP algorithm and other eight classical neural network algorithms.

## Data Availability

The data used to support the findings of this study are available from the corresponding author upon request.
